# Toxicity Evaluation of New Engineered Nanomaterials in Zebrafish

This article has been retracted.

**DOI:** 10.3389/fphys.2016.00130

**Published:** 2016-04-13

**Authors:** Maria V. Brundo, Roberta Pecoraro, Fabio Marino, Antonio Salvaggio, Daniele Tibullo, Salvatore Saccone, Vincenzo Bramanti, Maria A. Buccheri, Giuliana Impellizzeri, Viviana Scuderi, Massimo Zimbone, Vittorio Privitera

**Affiliations:** ^1^Department of Biological, Geological and Environmental Science, University of Catania Catania, Italy; ^2^Department of Chemical, Biological, Pharmaceutical and Environmental Sciences, University of Messina, Polo Universitario dell'Annunziata Messina, Italy; ^3^Experimental Zooprophylactic Institute of Sicily Catania, Italy; ^4^Department of Biomedical and Biotechnology Sciences, University of Catania Catania, Italy; ^5^CNR-IMM MATIS Catania, Italy

**Keywords:** *Danio rerio*, nanoparticles, nanomaterials, metallothioneins, zebrafish embryo toxicity test

## Abstract

The effect of the nanoparticles on the marine organisms, depends on their size, chemical composition, surface structure, solubility and shape. In order to take advantage from their activity, preserving the surrounding environment from a possible pollution, we are trying to trap the nanoparticles into new nanomaterials. The nanomaterials tested were synthesized proposing a ground-breaking approach by an upside-down vision of the Au/TiO_2_ nano-system to avoid the release of nanoparticles. The system was synthesized by wrapping Au nanoparticles with a thin layer of TiO_2_. The non-toxicity of the nano-system was established by testing the effect of the material on zebrafish larvae. *Danio rerio* o zebrafish was considered an excellent model for the environmental biomonitoring of aquatic environments and the Zebrafish Embryo Toxicity Test (ZFET) is considered an alternative method of animal test. For this reason zebrafish larvae were exposed to different concentrations of nanoparticles of TiO_2_ and Au and new nanomaterials. As biomarkers of exposure, we evaluated the expression of metallothioneins by immunohistochemistry analysis and western blotting analysis also. The results obtained by toxicity test showed that neither mortality as well as sublethal effects were induced by the different nanomaterials and nanoparticles tested. Only zebrafish larvae exposed to free Au nanoparticles showed a different response to anti-MT antibody. In fact, the immunolocalization analysis highlighted an increase of the metallothioneins synthesis.

## Introduction

Nanotechnology is the engineering of functional systems at the atomic, molecular, and supramolecular scale. The research field of Nanoparticle is currently an area of intense scientific interest due to a wide variety of potential applications in biomedical fields. In the nanotechnology field, a particle is defined as a small object that behaves as a whole unit with respect to its transport and properties. Nanoparticles (NPs) are particles between 1 and 100 nanometers (EU, 2011) in size and they have great scientific interest because they represent a bridge between bulk materials and atomic or molecular structures. The interesting and sometimes unexpected properties of nanoparticles are largely due to the large surface area of the material, which dominates the contributions made by the small bulk of the material.

It is well known that the major goals in designing nanoparticles as a delivery system are to control particle size, surface properties and release of pharmacologically active agents in order to achieve the site-specific action of the drug at the therapeutically optimal rate and dose regimen.

Wide dissemination of NPs is due to their physicochemical properties compared to fine particles (FPs) of the same composition.

A lot of nanoparticles are traditionally considered as chemically inert and biocompatible, in particular, titanium dioxide (TiO_2_) and gold (Au) nanoparticles (NPs) were identified as valuable tools in several research areas (Gerber et al., 2013; Liu and Ye, 2013).

TiO_2_ NPs are commonly-used due to their stronger catalytic activity when compared to TiO_2_ FPs. This increment of their catalytic activity was related to their smaller sizes, which allowed for larger surface area per unit mass. Some concerns have been also raised because these same properties of TiO_2_ NPs may present unique bioactivity and challenges to human health (Maynard and Kuempel, 2005; Tsuji et al., 2006).

Gold nanoparticles have been established as valuable tools in several areas of biomedical research. But in contrast to the multitude of studies that addressed the clinical use of gold nanoparticles, only little is known about potential toxicological effects of this NPs (Gerber et al., 2013).

In order to reduce the risk that the massive use of NPs can cause, it would be useful to fix them on substrates that allow to maintain their properties, but at the same time preventing their release into the environment. The proposed method involves the development an innovative TiO_2_/Au nano-composite synthesized by sputtering and atomic layer deposition (ALD) techniques. The peculiarity of this system is the wrapping of gold nanoparticles (~8 nm mean diameter) with a thin layer of TiO_2_ (~4 nm thick) (Scuderi et al., 2014). The ALD technique is one of the few techniques able to realize films with a controlled thickness of few nanometers. This effectively contributes to the photoreactions, avoiding any wastage of the material. This optimized design takes advantage on the presence of metal nanoparticles (in terms of electron trapping), without losing any TiO_2_ exposed surface. In addition, the form of thin film eliminates the problem of the particle filtration step after the water treatment.

The aim of present investigation is to evaluate the toxicity of the nano-composite by zebrafish embryo toxicity test (ZFET), an alternative method to animal testing, because embryos are not considered animals according to valid EU legislation (EC, 1986). ZFET represent an alternative approach to acute toxicity testing, since with the same sensitivity and specificity is possible to find more simplification, economicity, speedy of execution, as well as suggested by the European Community in order to decrease the impact of the experimental tests on live animals. The FET test is included in the guidelines to perform toxicity test about FDA and ICH for the pharmaceutical products and about EPA and OECD for the chemical substances (2013).

The purpose of this test is to determine the effects of chemicals on the embryonic stages of zebrafish. As biomarkers of exposure, we analyzed metallothioneins (MTs). MTs are a group of low molecular mass (2–16 kDa) single-chain proteins. They have low molecular weight, cysteine-rich, heavy metal binding proteins, shown to be involved in heavy metal ion homeostasis and detoxification (Kägi et al., 1984; Hamer, 1986; Kägi and Schaffer, 1988; Schroeder and Cousins, 1990; Suzuki et al., 1993; Ruttkay-Nedecky et al., 2013). Based on their affinity to metals these proteins are able to transport essential metals to place of need or detoxify toxic metals to protect cells. For these reasons the MTs play a key role in the maintaining of metal homeostasis. In addition, the ZFET results performed on new synthesized material, was compared with free Au and TiO_2_ nanoparticles.

## Materials and methods

### Synthesis of nanomaterials and nanoparticles

A gold film, with a thickness of ~5 nm, was sputtered on a quartz substrates. Then, the samples were annealed at 600°C for 1 h in a conventional furnace under a controlled N_2_ flux, in order to induce the self-organization of the metal nanoparticles. The as-synthesized gold nanoparticles (~8 nm in mean diameter) were covered with a thin layer of TiO_2_ (~4 nm in thickness), deposited by ALD (George, 2010). The ALD was performed with a Beneq TFS-200 system, with TiCl_4_ and de-ionized water as precursors, nitrogen as carrier gas, at a deposition temperature of 200°C. The deposition of the TiO_2_ film on top of the gold nanoparticles avoided the photocatalytic efficiency loss due to coverage of the TiO_2_ surface by the metal particles (Arabatzis et al., 2003; Armelao et al., 2007). This sample typology will be hereafter called “TiO_2_/Au” (i.e., TiO_2_ on Au nanoparticles). Another sample typology was synthesized: Au nanoparticles on top of TiO_2_ film (~4 nm in thickness), realized by ALD and sputtering, on a quartz substrate, that is the configuration commonly reported in the literature (Arabatzis et al., 2003; Armelao et al., 2007), hereafter called “Au/TiO_2_” (i.e., Au nanoparticles on top of the TiO_2_).The toxicity of free Au nanoparticles in salt water solution was also tested in order to discriminate the eventual impact of the stable nano-composite and of free nanoparticles. The Au nanoparticles were synthesized by pulsed laser ablation in liquid method. Dynamic light scattering technique evidenced a hydrodynamic diameter of the gold nanoparticles of 30 ± 2 nm.

### SEM analysis (day 0/day 12)

The structural characterization of the nanostructured materials was performed by scanningelectron microscopy (SEM). The analyses, in plan-view, were acquired by a field emission Zeiss Supra 25 microscope. The size distribution of the gold nanoparticles, deposited on the surface of the TiO_2_ film, was calculated by using the Digital Micrograph program by Gatan. In particular, several micrographs were taken into account, each of about 1700 × 1200 nm in size, containing ~2000 nanoparticles. The structural characterization and the relative gold nanoparticles distribution were performed before and after a 12 days dipping in aquatic environment, in order to evaluate the stability of the gold nanoparticles.

### Toxicity evaluation

#### Zebrafish maintenance and embryo collection

Zebrafish of the AB strain (wild-type) were obtained from the Center of Experimental Ichthyiopathology of Sicily (CISS), University of Messina, Italy, where they were kept in a “Fish facility” (Stand Alone Unit, Tecniplast), with a closed-loop system that allows the continuous monitoring of vital parameters. They were raised on a circulating aquarium system in an environmentally controlled room (28°C, 80% humidity), with the photoperiod adjusted to a 14 h light/10 h dark cycle. The larval and adult zebrafish were fed with brine shrimp (hatched from eggs in 10 mL in 2 L salt water) daily. For experiments, fertilized eggs were collected and chosen under a stereomicroscope (Leica M0205C, Multifocus) within 4 h post-fertilization (hpf). All embryos were derived from the same spawns of eggs.

#### Fish embryo toxicity (FET) test

Fish Embryo Toxicity (FET) test was effectuated according to OECD (2013) and ISO 15088. Zebrafish embryos exposed to “TiO_2_/Au” and “Au/TiO_2_” nanomaterials, to freeAu and TiO_2_NPs at different concentrations (10^9^, 10^10^, and 10^11^ in 5 ml of freshwater) for 4–96 hpf were measured for toxic effects of a continuing observation period. The experiment on nanomaterials was carried out on the material just produced (day 0) and then placed for 12 days (day 12) in water on an orbital shaker. The TiO_2_ and Au solutions were renewed and embryonic/larval mortality and hatching rate were evaluated every 24 h. Healthy embryos were placed in 24-well culture plates (10 embryos in 2 ml solution/well). Each group had five replicate wells. Each experiment was replicated four times. During the exposure period (4–96 hpf), photographs of the embryos were captured under a stereomicroscope (Leica M0205C, Multifocus) and the percentage of abnormal embryos was counted every 24 h.

#### Immunohistochemical analysis

Some larvae were used for immunodetection of biomarkers by immunofluorescence. Non-specific binding sites for immunoglobulins were blocked by incubations for 1 h with normal goat serum (Vector Laboratories) in PBS (1:10).

The larvae were incubated overnight in a humid chamber at 4°C with the primary antibody anti-mouse-MT (1:500, Abcam). After a rinse in PBS for 10 min, the samples were incubated for 2 h at room temperature with fluorescein isothiocyanate (FITC) conjugated goat anti-mouse IgG (Sigma).

Negative controls for immunohistochemical labeling were performed by substitution of blank sera (without antibodies) for the primary antisera. Observations were carried out using confocal laser scanning microcopy (CLSM; Zeiss LSM 700), equipped with the ZEN-2011 software and with a green fluorescence filter set.

#### Western blotting analysis

MTs determination in larvae was carried out by Western blotting analysis. The samples were weighed, homogenized 1:10 (w/v) in a lysis buffer (Tris–HCl 40 mM, EDTA 25 mM, 0.2% SDS, pH 7.4) containing 1/100 (v/v) protease inhibitors (Sigma) and centrifuged. Total protein concentration in the supernatant was determined according to the Bradford method (Bradford, 1976). Thirty micro gram of protein/lane was analyzed by minigel SDS-PAGE and transferred to a nitrocellulose membrane using Transblot (Biorad). The proteins levels were measured by incubating nitrocellulose membranes overnight at 4°C with mouse monoclonal primary antibody anti-MTs (1:500, Abcam, ab57287). The complex protein-primary antibody was detected using a HRP-conjugated Ig-G anti-mouse secondary antibody (1:1000, Abcam) by chemiluminescent method. Blots were scanned and quantified by a specific software (Image J).

#### Gene expression analysis

RNA was extracted by Trizol reagent (Invitrogen, Carlsbad, CA, USA). First strand cDNA was then synthesized with Applied Biosystem (Foster City, CA, USA) reverse transcription reagent. Mt mRNA expression was assessed using a fuorescence-based real-time detection method by 7900HT Fast Real Time PCR System (Life technologies, Carlsbad, CA, USA). For each sample, the relative expression level of mt (forward primer 5′-GCC AAG ACT GGA ACT TGC AAC-3′; reverse primer 5′-CGC AGC CAG AGG CAC ACT-3′; amplicon sizeis 130 bp) mRNA was normalized using β-actin (forward primer 5′-CTT GGG TAT GGA ATC TTG CG-3′; reverse primer 5′-AGC ATT TGC GGT GGA CGA T-3′; amplicon sizeis 88 bp) as an invariant control.

#### Statistical analysis

Statistical analysis was performed with Prism Software (Graphpad Software Inc., La Jolla, CA, USA). Data were expressed as mean or SD. Statistical analysis was carried out by unpaired *t*-test or ANOVA testto compare the means of more than two samples. The significance of differences between means was analyzed by ANOVA. *P* < 0.05 was considered statistically significant between experimental and control groups.

## Results

### SEM analysis

SEM images of the Au nanoparticles on the TiO_2_ film show that before the immersion (Figure 1A) the samples consisted of a homogeneous distribution of gold nanoparticles with a TiO2 coverage about ~36%. After 21 days in aquatic environment, the analyses indicated a reduction of the TiO2 coverage about ~36–28% (Figure 1B). Thus, the liquid environment induced detachment of the Au nanoparticles from the TiO_2_ underneath film. The same investigation was done with the samples with the TiO_2_ film on top of the gold nanoparticles. In this case, the SEM analyses showed the same gold distribution, before and after the 12 days dipping, indicating a strong stability of the embedded AuNPs.

**Figure 1:** **SEM Images nanomaterials**. Nanocomposed of Au nanoparticles on TiO_2_ flat film **(A)** before and **(B)** after a 12 days dipping in aquatic environment.

### Fish embryo toxicity (FET) test

Fish Embryo Toxicity test showed that neither mortality nor sublethal effects were caused by the different nanomaterials and free nanoparticles tested. In particular, the following different endpoints were evaluated: viability, growth (larval length), brain morphology, pharyngeal arches and jaw, other craniofacial structures, heart, fins, notochord, somites, tail, body shape, cardiovascular function, yolk sac and locomotor function and touch response.

### MTs analysis

The NMs (“TiO_2_/Au” and “Au/TiO_2_”) were immersed in water until 12 days in agitator. The Zebarfish larvae were added to aquatic sample the first day (Time 0) or after 12 (Time 12) days for 96 hpf. Immunohistochemical analysis performed in larvae exposed to “TiO_2_/Au,” “Au/TiO_2_” in aquatic samples at Time 0 and Time 12, and free TiO_2_, showed the presence of MTs only in head region (Figure 2A), as well as to control samples (untreated). Moreover, the zebrafish exposed to AuNPs showed a positive response to anti-MT in whole body (Figure 2B). In addition, we evaluated the mRNA and protein expression of MTs. We observed that the free TiO_2_, TiO_2_/Au and Au/TiO_2_ did not able to induce the mt mRNA expression, while free Au increased mt levels of about 20-fold (*p* < 0.0001) respect to untreated sample. This result was confirmed by western blotting analysis (Figures 3, 4A,B).

**Figure 2:** **Larvae zebrafish 96 hpf treated with anti-MT antibody. (A)** Larvae exposed to free TiO_2_ showed the presence of MTs only in head region. Same result was shown in the control samples and in the larvae exposed to “TiO_2_/Au,” “Au/TiO_2_”at Time 0 and Time 12. **(B)** Zebrafish exposed to Au NPs showed a positive response to anti-MT in whole body. Scale bar: 150 μm

**Figure 3:** **Western blotting analysis for evaluation the effects of exposure to nanomaterials**. The MTs level, in untreated samples and in larvae exposed to nanomaterials before (Time 0) and after a 12 days (Time 12) dipping in aquatic environment was evaluated. The data are expressed as mean ± SEM. Statistical analysis was carried out by ANOVA test. A *p*-value of less than 0.05 (*p* < 0.05) was accepted as statistically significant between experimental and control groups.

**Figure 4:** **(A)** Western blotting analysis for evaluation the effects of exposure to free nanoparticles and nanomaterials. The MTs level in untreated samples and in larvae exposed to nanomaterials (Time 0/Time12) and free TiO_2_ and Au nanoparticles was evaluated. The data are expressed as mean ± SEM. Statistical analysis was carried out by ANOVA test. A *p*-value of less than 0.05 (*p* < 0.05) was accepted as statistically significant between experimental and control groups. **(B)** mRNA gene expression of mt in zebrafish after exposure to free nanoparticles and nanomaterials. The mt mRNA expression was increased only in free Au treatment. *Bars* represent the mean ± SEM of three independent experiments. ***P < 0.0001 vs. untreated sample. (Calculated value of 2^∧^−ΔΔ Ct in untreated sample was 1).

## Discussion

The toxicology of engineered NMs is a relatively new and evolving field and although the their applications are increasing, there are many concerns about their environmental and health impacts (Asharani et al., 2008). Alarge number of studies carried out on AuNPs have produced conflicting results. In fact, despite continuous attempts to establish a correlation between structure of the particles and their interactions with biological systems, we are still far from elucidating with certainty the toxicological profile of AuNPs (Fratoddi et al., 2015). Among these investigations, a large numbers of authors has confirmed the non-toxicity of AuNPs (Dobrovolskaia and McNeil, 2007; Patra et al., 2007; Cho et al., 2009; Peng et al., 2009; Tedesco et al., 2010), conversely, others have observed the toxicity of AuNPs (Pan et al., 2007; Zhang et al., 2009; Sung et al., 2011).

Despite, some authors showed low toxicity of others particles such as TiO2 NPs (ACGIH, 1992; Participants IRSIW, 2000), several studies demonstrated that exposure to high concentrations of TiO_2_ particles was able to induce lung tumors formation after 2 years in rats (Lee et al., 1985). Moreover, the International Agency for Research on Cancer (IARC), has classified TiO_2_ as a possibly carcinogenic to human (Group 2B carcinogen) (IARC, 2010).

The proposed method involves the development of an innovative nanomaterial that could help to overcome problems related to the toxic effects of NPs, being able to exploit all their qualities.

In our study we used zebrafish, as animal model, because it has been recommended by some researches as an inexpensive, quick and easy model to assess the NMs toxicity (Fako and Furgeson, 2009), and it can offer many advantages for toxicological research (Bourdineaud et al., 2013; Pecoraro et al., 2015). In particular, we have used ZFET, an alternative approach to acute toxicity testing, in order to decrease the impact of the experimental tests on live animals as well as suggested by the European Community.

As biomarkers of exposure, we analyzed metallothioneins (MTs). The use of MTs is supported by several studies. Some authors showed that MT proteins could be a potential biomarkers for metal contamination in aquatic environment (Benson et al., 1990; Couillard, 1997; AETE, 1999; Langston et al., 2002; De Domenico et al., 2011; Copat et al., 2012). Moreover, some studies demonstrated that during oogenesis the MTs level in zebrafish slowly decreases during the early stages of development (Riggio et al., 2003; Chen et al., 2004). In particular, they demonstrated a gradual decrease in the level of MT transcripts during the early embryonic stages (Chen et al., 2004). Chen et al. (2002) also observed a strong ubiquitous expression of metal-responsive transcription factor (MTF-1), the responsible for Mt gene expression (Günes et al., 1998). Furthermore, the expression patterns of MT (Chen et al., 2004) and MTF-1 (Chen et al., 2002) at prim-5 stage are in opposite manner: the former expressed well in the tail region while the latter in head region. For this reason, the authors suggest that MT may be involved in urinary and digestive system whereas, MTF-1 not and the expression of MT in the tail region may be due to other regulatory factors. The MT expression pattern is more comparable with MTF-1, during early hatching period (Chen et al., 2004). In particular, after hatching, no significant MT signal could be observed in the tail region. On 1dph, clear as well as distinct MT expression signals are seen in common cardinal vein and chloride cells. The signals observed on 1dph at lateraland dorsal views become stronger on 2dph. The intensity of signals at common cardinal vein, pronephric region, and retina almost vanished on 3dph. The intensity of staining due to MT expression at cerebellum and pronephric region on 4dph becomes increased and maintains until 12dph, show that MT expression plays a role on zebrafish embryogenesis and early larval development (Chen et al., 2004).

In our experimental model, the MTs expression shows a high susceptibility to gold free metallic nanoparticles, highlighting the importance of their trapping inside the new engineered nanomaterials. This could be useful to make maximum use of potential of NPs removing the possible risk of damage the environment.

However, the synthesized material with Au nanoparticles on top, showed a dispersion of Au nanoparticles in the liquid environment, due to their instability in the aqueous solution that clearly represents an environmental contamination issue. For this reason, in the next future, the nanometric TiO_2_ wrapping of Au nanoparticles could have a great potential as eco-friendly materials.

## Author contributions

MVB and RP have carried out the planning of experiments, have elaborated the data and have drafted the manuscript; RP has carried out experiments on zebrafish larvae; RP and DT have carried out experiments of western blotting, immunohistochemical analysis and gene expression analysis; VP, FM, AS, and MAB have participated in conceiving and designing the study and have revised the manuscript; SS has made confocal analysis; VS has made SEM analysis; GI, has realized NMs; MZ has realized NMs; VB have revised the manuscript.

## Funding

This work has been supported by the VII FP project Winning Applications of nanoTEchnologies for Resolutive hydropurification (WATER) funded by the European Commission (Grant 316082).

### Conflict of interest statement

The authors declare that the research was conducted in the absence of any commercial or financial relationships that could be construed as a potential conflict of interest.
